The article "The Impact of Charlson Comorbidity Index on Mortality From SARS-CoV-2 Virus Infection" was retracted in 2022. Reasons: false authorship; lack of ethics approval or compliance; concerns about the data; concerns about the authorship.

# The Impact of Charlson Comorbidity Index on Mortality From SARS-CoV-2 Virus Infection

**DOI:** 10.7759/cureus.19937

**Published:** 2021-11-27

**Authors:** Jawad Ahmed, Camilo Andrés Avendaño Capriles, Natalia M Avendaño Capriles, Shivani M Mehta, Nattaliea Khan, Sheharyar Tariq, Ramsha Abbas, Sohaib Tousif, Khizer Shamim

**Affiliations:** 1 Medicine, Liaquat National Hospital and Medical College, Karachi, PAK; 2 Foundations of Clinical Research (FCR) Program, Harvard Medical School, Boston, USA; 3 Medicine, Universidad del Norte, Barranquilla, COL; 4 Medicine, Xavier University School of Medicine, Oranjestad, ABW; 5 Medicine, Ziauddin University, Karachi, PAK; 6 Medicine, Lahore Medical and Dental College, Lahore, PAK; 7 Medicine, Shifa College of Medicine, Islamabad, PAK; 8 Medicine, Ziauddin Medical University, Karachi, PAK; 9 Medicine, Ziauddin University Hospital, Karachi, PAK

**Keywords:** mortality, impact, covid-19, colacd, charlson comorbidity index

## Abstract

Introduction: Charlson Comorbidity Index (CCI) is a simple, validated, and readily acceptable method of determining the risk of mortality from comorbid disease. It has been used as a predictor of long-term survival and prognosis. The aim of this study is to determine the impact of CCI score on mortality in COVID-19 hospitalized patients and test the efficacy of the CoLACD score (COVID-19 lymphocyte ratio, age, CCI score, dyspnoea) in predicting mortality among hospitalized COVID-19 patients.

Methodology: It was a retrospective cohort, and the data of this study were gathered from two tertiary hospitals of Karachi, including Liaquat National Hospital and Ziauddin Hospital. Data of patients hospitalized in any of these tertiary care hospitals and diagnosed with confirmed COVID-19 infection were used in the study from January 15, 2021, to April 30, 2021.

Results: The mean age of participants was 53.22 (±14.21) years. The majority of participants were males (74.91%). Predictors of mortality include CCI score, age of participants, D-dimer, smoking status, and shortness of breath. The sensitivity of this CoLACD score was 80.23%, and specificity was 50.23% (diagnostic accuracy is 60.45%). The negative predictive value (NPV) of this test was 39.44%, and the positive predictive value (PPV) was 83.01%.

Conclusion: Our study showed that CCI can be used in a clinical setting to achieve a prediction of mortality in COVID-19 patients.

## Introduction

Coronavirus disease (COVID-19) first emerged in Wuhan, China, in December 2019, and since then, the number of confirmed cases and deaths has been rising globally. There have been around 240 million confirmed cases of COVID-19, including 4,927,723 deaths globally reported by the World Health Organization (WHO) [1]. It is well-established from descriptive observational studies that patients with comorbidities are disproportionately impacted by COVID-19 and have inferior clinical outcomes [2]. The first case of COVID-19 was reported in Pakistan on February 2021, and since then numerous cases of COVID-19 have been reported, and a large number of individuals have been hospitalized due to disease severity [3]. Thousands of individuals died as a result of the COVID-19 epidemic; therefore, early detection for severe cases is important.

Various studies have been conducted that determined the radiological, laboratory, epidemiological, clinical, and demographic characteristics of severe COVID-19 cases [4]. In the study conducted by Du et al. to determine the predictors of mortality for patients with COVID-19 pneumonia caused by SARS-CoV-2, it was found that older age, cerebrovascular disease, D-dimer levels are predictors of mortality [5]. In Pakistan, where the burden of COVID-19 is high, and the lack of effective health care facilities can delay management and care provided to critical patients, it is imperative to develop and test a simple scoring system to predict mortality predictors and determine disease severity for early management.

Multiple risk factors are associated with mortality in COVID-19 patients; therefore, only a single parameter will not be enough for predicting mortality in patients. That is why new scores have been developed for predicting COVID-19 severity, and many valid and well-known scores have been adapted nowadays for COVID-19, including NEW2 (National Early Warning Score), CURB-65 (confusion, uremia, respiratory rate, BP, age ≥ 65 years), qSOFA (quickSOFA), and MulBSTA (multilobular infiltration, hypolymphocytosis, bacterial coinfection, smoking history, hypertension, and age) [6]. These scores are either multi-parameter or require complex laboratory findings. Some of them necessitate math, and the components of the scores are difficult to recall. As a result, in the current pandemic situation, and with an understanding of the necessity of early diagnosis of severe patients, a simple score may be useful to the doctor. A simple hemogram parameter may be beneficial for guiding therapy and determining the course of the disease in the primary health settings without the requirement for a pulse oximeter by simply asking comorbidities, questioning the symptom, dyspnea [6].

A scoring model was developed by Ji et al. called a CALL (C = comorbidity, A = age, L = lymphocyte count, L = lactate dehydrogenase [LDH]) score to predict the severity of disease among COVID-19 patients [7]. This score was developed to estimate the risk of mortality utilizing four parameters, including LDH, lymphocyte number, age, and comorbidity. However, in this model, comorbidity was not specified, and studies have shown that certain morbidities, including diabetes, hypertension, cardiovascular disease, and respiratory disease can increase the risk of mortality among COVID-19 patients [6]. Therefore, in the novel CoLACD (CoVID19 lymphocyte ratio, age, CCI score [Charlson comorbidity index], dyspnoea) model developed by Varol et al., a verified comorbidity index CCI score was used [6].

CCI is a relatively simple and readily acceptable method of determining the risk of mortality from comorbid disease and has been utilized as a predictor of long-term survival and prognostic tool [8]. It was developed in 1987, and since then, it has been used in many studies [9]. It is believed that because the severity of COVID-19 is impacted by age and comorbidities, this simple index, along with reported symptoms and basic laboratory data, can be used to predict death in COVID-19-infected, hospitalized patients. Thus, the aim of this study is to determine the impact of CCI score on mortality in COVID-19 hospitalized patients and test the efficacy of the CoLACD score in predicting mortality among hospitalized COVID-19 patients.

## Materials and methods

It was a retrospective cohort, and the data of this study were gathered from two tertiary hospitals of Karachi, including Liaquat National Hospital and Ziauddin Hospital. For this retrospective, non-interventional, and multicenter case-cohort study, patients diagnosed with confirmed COVID-19 infection which hospitalized in the above tertiary care hospitals were enrolled in the study from January 15, 2021, to April 30, 2021. All patients had a nasopharyngeal swab test for the SARS-CoV-2 virus utilizing real-time reverse transcriptase-polymerase-chain-reaction technology (RT-PCR). Positive RT-PCR results from nasopharyngeal swab samples were considered laboratory-confirmed patients.

The patients’ data, including demographic data, smoking status, comorbidities, symptoms at the time of admission, laboratory parameters, and outcomes, were collected from the hospital management information system (HMIS). CCI was calculated from the HMIS. Two investigators reviewed the data and double-checked it independently. Patients with missing CCI scores were not included in the final analysis. CoLACD scores were computed based on four parameters, including age, lymphocytes %, CCI score, and shortness of breath. The calculation of the CoLACD score was based on points as shown in Table 1. CoLACD score of less than 2.5 was considered as a lower risk of mortality, while a score of more than 2.5 was categorized as high mortality risk. The cut-off was adopted from the study conducted by Varol et al. [6].

**Table 1:** Calculation of CoLACD CoLACD: CoVID-19 lymphocyte ratio, age, CCI score, dyspnoea

	Points
Lymphocytes %	
≥17.6	0
<17.6	1
Age (years)	
<50	0
50-65	1
≥65	2
CCI score	
≥3	1
<3	0
Dyspnoea	
With	1
Without	0

Statistical analysis

Data analysis was done using STATA version 16.0 (StataCorp, College Station, TX). Continuous variables were presented with their mean and standard deviation, while frequency and percentage were presented for categorical variables. To determine the impact of different independent variables with mortality, t-test and chi-square test of independence were used for continuous and categorical variables, respectively, and variables significant in this step will be used in multivariable logistic regression. P-value <0.05 was considered statistically significant. To assess the impact of CCI score on the mortality of patients, multivariable logistic regression was used to adjust for confounding variables. To assess the predicting performance of CoLACD score, sensitivity, specificity, positive predictive value (PPV) and negative predictive value (NPV), and diagnostic accuracy were calculated using outcome (death vs. alive) as a gold standard.

## Results

From January 16, 2021, to May 21, 2021, 610 patients were admitted to two tertiary care hospitals of Karachi with confirmed COVID-19 infection confirmed by polymerase chain reaction testing from nasopharyngeal samples. After excluding patients who did not fulfill the exclusion criteria, data of 552 patients were included in the final analysis. The mean age of participants was 53.22 (±14.21) years. The majority of participants were males (74.91%). As per the disease severity, the majority of patients had moderate severity (32.69%), while the same number of patients had a critical disease. Comorbidities associated with mortality including diabetes (p-value<0.001) and chronic lung disease (p-value<0.001).

The characteristics of survivors and deceased are shown in Table 1. Age is significantly different between survivors and deceased (p-value=0.001). In survivors, the mean age is 50.19 (±13.76) years that is significantly lesser as compared to the deceased patients (59.19 [±14.05] patients). When we compared the symptoms of patients at the time of presentation, only dyspnea was significantly different between the two groups (p-value=0.047), as shown in Table 2. The proportion of critical patients were higher in a deceased group (59.32%) as compared to the survivor group (20.57%), and the difference was significant between the two groups (p-value=0.001).

**Table 2:** Comparison of demographic and clinical findings of COVID-19 patients who died and survived *Significant at p-value<0.05 ^Mean (standard deviation)

Variables	Survivors n(%)	Deceased n(%)	P-value
Age of patients	50.59 (13.76)	59.19 (14.05)	0.001*
Gender			
Male	283 (72.75)	141 (79.66)	0.079
Female	106 (27.25)	36 (20.34)	
Charlson Comorbidity Index			
Mild	81 (20.82)	7 (3.95)	0.001*
Moderate	157 (40.36)	28 (15.82)	
Severe	71 (18.25)	37 (20.90)	
Critical	80 (20.57)	105 (59.32)	
Smoking Status			
Non-smoker	310 (79.69)	110 (62.15)	0.001*
Ex-smoker	53 (13.62)	29 (16.38)	
Active smoker	26 (6.68)	38 (21.47)	
Symptoms at the time of admission			
Fever	302 (77.63)	140 (79.10)	0.152
Cough	240 (61.70)	126 (71.19)	0.201
Dyspnea	277 (71.21)	145 (81.92)	0.047*
Runny nose	28 (7.20)	5 (2.82)	0.277
Sore throat	21 (2.40)	4 (2.26)	0.644
Diarrhea	25 (6.42)	8 (4.51)	0.251
Chills	35 (8.99)	12 (6.78)	0.181
Nausea and vomiting	8 (2.05)	6 (3.38)	0.462
Fatigue	12 (3.08)	10 (5.64)	0.388
Loss of smell	210 (53.98)	90 (50.84)	0.349
Loss of taste	170 (43.70)	83 (46.89)	0.155
Comorbidities			
Diabetes	121 (33.80)	95 (57.93)	0.001*
Hypertension	165 (42.41)	85 (42.02)	0.069
COPD/asthma	132 (36.87)	85 (51.83)	0.001*
Renal disease	20 (5.59)	19 (11.59)	0.109
Active malignancy	9 (2.32)	6 (3.39)	0.299
Liver disease	5 (1.28)	4 (2.26)	0.284

Laboratory findings

Platelet count and blood urea nitrogen (BUN) were statistically significant between the two groups (Table 3). Other laboratory findings that were significantly different between the two groups included serum albumin, serum LDH, serum C-reactive protein (CRP), and serum D-Dimer. Overall, 72% of participants had abnormal findings on the X-ray, and the difference of abnormal findings was insignificantly different in the two groups (p-value=0.133).

**Table 3:** Comparison of laboratory findings of COVID-19 patients who died and survived *Significant at P-value<0.05 ^n (%) BUN: blood urea nitrogen, ALT: alanine transaminase, LDH: lactate dehydrogenase, CRP: C-reactive protein

Laboratory parameter	Survivors (mean±SD)	Deceased (mean±SD)	P-value
Hemoglobin (g/dl)	12.31±2.99	12.67±2.36	0.171
Hematocrit	36.54±7.67	35.86±7.95	0.367
Total WBC count (×10^9^/L)	17.67±5.23	13.40±6.88	0.161
Lymphocytes (%)	12.72±7.63	11.80±8.72	0.215
Platelet count (×10^9^/L)	259.55±186.21	252.55±125.55	0.041*
BUN (mg/dl)	18.10±13.50	26.09±18.23	0.001*
Creatinine (mg/dl)	1.50±0.79	1.63±1.07	0.322
Sodium (mEq/L)	135.58±7.29	135.93±5.48	0.574
Potassium(mEq/L)	4.22±0.58	4.18±0.56	0.441
Total bilirubin (mg/dL)	0.72±0.61	0.67±0.41	0.185
ALT (U/L)	55.75±41.36	77.76±57.08	0.041
Serum ferritin (ng/ml)	1098.95±1172.38	1192.99±871.63	0.347
Serum albumin (g/dl)	3.39±0.48	3.06±0.59	0.001*
Serum LDH (U/L)	507.48±408.85)	672.06±439.67	0.001*
CRP (MG/L)	130.06±90.05	184.01±121.02	0.001*
Troponin I levels (ng/L)	80.88±393.95	108.80±229.93	0.398
D-dimer (ng/ml FEU)	3292.98±4695.17	5761.97±5772.98	0.001*
Abnormal X-ray findings^	286 (73.52)	121 (68.36)	0.133

Predictors of mortality

To determine the factors associated with mortality, multivariable logistic regression was used including all variables significant at univariate analysis, and significant variables are shown in Table 4. It was found that odds of death are 6.82 times greater in severe patients and 13.16 times greater in critical patients than mild patients (p<0.001). Likewise, increased age is significantly associated with increased odds of mortality (AOR=1.05, p-value=0.001). Third, in smokers, the odds of mortality are 3.01 times greater than non-smokers (p-value=0.001). Patients having dyspnea had 1.83 times higher mortality risk compared with patients without dyspnea (p-value=0.01). Lastly, patients with increased D-dimer are at greater risk of mortality (AOR=1.06, p-value=0.001).

**Table 4:** Multivariate logistic regression analysis of mortality risk factors for patients with COVID-19 CI: confidence interval

Variable	Categories	AOR	95% CI	P-value
Charlson Comorbidity Index	Mild	Ref		
	Moderate	2.03	0.82–4.99	0.121
	Severe	6.82	2.71–17.16	0.001
	Critical	13.16	5.44–31.84	0.001
Age of patients		1.05	1.03–1.07	0.001
Smoking status	Non-smoker	Ref		
	Ex-smoker	0.87	0.43–1.73	0.497
	Active smoker	3.01	1.56–5.76	0.001
D-dimer		1.06	1.02–1.12	0.001
Shortness of breath	No	Ref		
	Yes	1.83	1.17–2.84	0.007

CoLACD scoring model

To test the sensitivity and specificity of the CoLACD scoring model, the score was compared with the outcome. The sensitivity of this score was 80.23%, and specificity was 50.23% (diagnostic accuracy is 60.45%). The negative predictive value of this test was 39.44%, and the positive predictive value was 83.01%. The risk of mortality was 3.18 times higher in patients with a CoLACD mortality score higher than 2.5 points than patients with a score lower than 2.5 (OR = 3.18; 95% CI 2.08-4.84; P<0.001).

## Discussion

In past studies, it has been shown that comorbidities play an important role in hospitalized COVID-19 patients. CCI is a valid and reliable tool to predict mortality, but its impact on COVID-19 has not been explored properly. The study conducted by Varol et al. found that high comorbidity index increases the likelihood of mortality 10.7 times [6]. Similar findings were also reported in our study which found that the likelihood of mortality was high in severe and critical patients.

Several studies have determined the factors associated with poor prognoses such as age, lymphocytes, comorbidities, and different laboratory parameters, including IL-6, dehydrogenase dimer, lactate, cardiac troponin, and serum ferritin [5,10]. Several biomarkers like ferritin, procalcitonin, CRP, and D-dimer are usually elevated in severe COVID-19 cases, and these laboratory parameters can be used to predict outcomes in severe COVID-19 patients. In our study, D-dimer was associated with mortality among COVID-19 patients [11].

A study conducted by Yonas et al. has found that during the COVID-19 pandemic, mortality is also predicted by gender, the presence of certain comorbidities like respiratory diseases, cerebrovascular diseases, cardiovascular diseases, and diabetes can increase the risk of mortality among hospitalized COVID-19 patients [12]. Iman et al. have also found that multiple comorbidities are independent risk factors of mortality among COVID-19 patients [13]. In the current study, mortality was higher among patients with certain comorbidities, including diabetes and respiratory diseases. Our study has also found that increased age is associated with higher chances of mortality among COVID-19 patients. However, no significant association was found between gender and mortality. Past studies have also found an association between age and mortality [8,14].

The current study has tested the efficacy of CoLACD score in COVID-19 hospitalized patients. Our study has tested its effectiveness in the Pakistani population. As per Varol et al. study, the sensitivity and specificity of this score are 82% and 73% specificity [8]. By using the same cut-off, the sensitivity of this score was 80.23%, and specificity was 50.23% in the current study. In addition, it has also been found in our study that the risk of mortality was greater in patients with a CCLAD score of more than 2.5 points than patients with a score lower CoLACD score. Similar findings were also reported in the previous research [6].

In the case of the COVID-19 outbreak, CCI scoring can be particularly beneficial in predicting the requirement for intensive care unit (ICU) admission, respiratory support, or the likelihood of hospital readmission [15]. Patients with comorbidities are more likely to develop acute cardiovascular illnesses; nonetheless, while COVID-19 in these patients is worrying, it should not preclude or delay appropriate treatment [16]. Knowing the clinical characteristics of patients and risk factors that predict poor outcomes in COVID-19 transmission is critical for planning thorough treatment and dedicating vital resources as the pandemic continues to spread over the world.

The current study has certain limitations. First, the data were only obtained from two tertiary care hospitals in Karachi, and we included only COVID-19 patients hospitalized for COVID-19 in the first quarter of 2021. Second, as this was a retrospective study, many laboratory parameters such as ferritin and D-dimer were missing in some patients. However, components that were required to calculate CoLACD scores were completed in HMIS. 

## Conclusions

In conclusion, our study found that CCI score is associated with a great likelihood of mortality in COVID-19 hospitalized patients. Other factors significantly associated with mortality included age, D-Dimer, and shortness of breath. This study adopted a CoLACD score that is based on routine laboratory tests. These tests are done in first-line health settings to predict mortality among patients with COVID-19. Considering the simplicity of this tool, if this can be validated in prospective studies, the CoLACD score can be utilized for efficient use of medical resources in the COVID-19 pandemic, particularly in hospitals with limited resources.

## References

[1] Marroquín B, Vine V, Morgan R (2020). Mental health during the COVID-19 pandemic: effects of stay-at-home policies, social distancing behavior, and social resources. Psychiatry Res.

[2] Christensen DM, Strange JE, Gislason G, Torp-Pedersen C, Gerds T, Fosbøl E, Phelps M (2020). Charlson comorbidity index score and risk of severe outcome and death in Danish COVID-19 patients. J Gen Intern Med.

[3] Ilyas N, Azuine RE, Tamiz A (2020). COVID-19 pandemic in Pakistan. Int J Transl Med Res Public Health.

[4] Li X, Xu S, Yu M (2020). Risk factors for severity and mortality in adult COVID-19 inpatients in Wuhan. J Allergy Clin Immunol.

[5] Du RH, Liang LR, Yang CQ (2020). Predictors of mortality for patients with COVID-19 pneumonia caused by SARS-CoV-2: a prospective cohort study. Eur Respir J.

[6] Varol Y, Hakoglu B, Kadri Cirak A (2021). The impact of charlson comorbidity index on mortality from SARS-CoV-2 virus infection and A novel COVID-19 mortality index: CoLACD. Int J Clin Pract.

[7] Ji D, Zhang D, Xu J (2020). Prediction for progression risk in patients with COVID-19 pneumonia: the CALL score. Clin Infect Dis.

[8] Carter JH, Sketris IS, Tamim H, Levy AR, Langley JM (2019). Determining proton pump inhibitor prescription dispensing patterns and adherence to STOPP criteria for Nova Scotia Seniors Pharmacare Program beneficiaries. J Popul Ther Clin Pharmacol.

[9] Charlson ME, Pompei P, Ales KL, MacKenzie CR (19871). A new method of classifying prognostic comorbidity in longitudinal studies: development and validation. J Chronic Dis.

[10] Chen N, Zhou M, Dong X (2020). Epidemiological and clinical characteristics of 99 cases of 2019 novel coronavirus pneumonia in Wuhan, China: a descriptive study. Lancet.

[11] Huang I, Pranata R, Lim MA, Oehadian A, Alisjahbana B (2020). C-reactive protein, procalcitonin, D-dimer, and ferritin in severe coronavirus disease-2019: a meta-analysis. Ther Adv Respir Dis.

[12] Yonas E, Alwi I, Pranata R (2021). Effect of heart failure on the outcome of COVID-19 - a meta analysis and systematic review. Am J Emerg Med.

[13] Imam Z, Odish F, Gill I (2020). Older age and comorbidity are independent mortality predictors in a large cohort of 1305 COVID-19 patients in Michigan, United States. J Intern Med.

[14] Gong J, Ou J, Qiu X (2020). A tool for early prediction of severe coronavirus disease 2019 (COVID- 19): a multicenter study using the risk nomogram in Wuhan and Guangdong, China. Clin Infect Dis.

[15] Wang D, Hu B, Hu C (2020). Clinical characteristics of 138 hospitalized patients with 2019 novel coronavirus-infected pneumonia in Wuhan, China. JAMA.

[16] Myrstad M, Ihle-Hansen H, Tveita AA, Andersen EL, Nygård S, Tveit A, Berge T (2020). National Early Warning Score 2 (NEWS2) on admission predicts severe disease and in-hospital mortality from Covid-19 - a prospective cohort study. Scand J Trauma Resusc Emerg Med.

